# Empirical Method for Thyroid Disease Classification Using a Machine Learning Approach

**DOI:** 10.1155/2022/9809932

**Published:** 2022-06-07

**Authors:** Tahir Alyas, Muhammad Hamid, Khalid Alissa, Tauqeer Faiz, Nadia Tabassum, Aqeel Ahmad

**Affiliations:** ^1^Department of Computer Science, Lahore Garrison University, Lahore 54000, Pakistan; ^2^Department of Statistics and Computer Science, University of Veterinary and Animal Sciences, Lahore 54000, Pakistan; ^3^Saudi Aramco Cybersecurity Chair, Networks and Communications Department, College of Computer Science and Information Technology, Imam Abdulrahman Bin Faisal University, P.O. Box 1982, Dammam 31441, Saudi Arabia; ^4^Department of Enterprise Computing, Skyline University College, Sharjah, UAE; ^5^Department of Computer Science & Information Technology, Virtual University of Pakistan, Lahore 54000, Pakistan; ^6^University of Chinese Academy of Sciences (UCAS), Beijing, China

## Abstract

There are many thyroid diseases affecting people all over the world. Many diseases affect the thyroid gland, like hypothyroidism, hyperthyroidism, and thyroid cancer. Thyroid inefficiency can cause severe symptoms in patients. Effective classification and machine learning play a significant role in the timely detection of thyroid diseases. This timely classification will indeed affect the timely treatment of the patients. Automatic and precise thyroid nodule detection in ultrasound pictures is critical for reducing effort and radiologists' mistake rate. Medical images have evolved into one of the most valuable and consistent data sources for machine learning generation. In this paper, various machine learning algorithms like decision tree, random forest algorithm, KNN, and artificial neural networks on the dataset create a comparative analysis to better predict the disease based on parameters established from the dataset. Also, the dataset has been manipulated for accurate prediction for the classification. The classification was performed on both the sampled and unsampled datasets for better comparison of the dataset. After dataset manipulation, we obtained the highest accuracy for the random forest algorithm, equal to 94.8% accuracy and 91% specificity.

## 1. Introduction

Approximately about 4.6 percent of the population of ages 12 and greater suffers from hypothyroidism, and 1.2 percent of people in the USA have hyperthyroidism, equal to 1 out of 100 people. Machine learning is implemented in many fields today. But most significant improvements are made in the field of medicine. To detect thyroid disease, blood tests and medical imaging are performed (ultrasound). Awareness about thyroid disease is necessary as it will play a significant role in the early detection and curing of this problem. The thyroid is an organ in the human body. It produces the hormone required by the human body. The hormones travel in the bloodstream, and it affects the metabolism and growth of humans. It is located below Adam's apple. Thyroid functionality is used for the interpretation and diagnosis of the disease. The thyroid gland produces hormones that control the growth and metabolism used for the body's energy purposes. The thyroid gland also contributes to development in children and adults. The thyroid gland also maintains body temperature. Minor issues with the gland can cause a problem all over the body. The functionality of the thyroid gland and the test results conducted after taking a blood sample are used to signify if the thyroid gland is working correctly. This hormone's secretion tells whether the thyroid is producing too much hormone or too little hormone for proper function. The condition in which little thyroid hormone is produced is called hypothyroidism. When the hormone is too much, it is referred to as hypereuthyroidism. The thyroid gland produces two main hormones—triiodothyronine (T3) and thyroxine (T4).

Thyroid disorder is one of the most frequent illnesses among women. Thyroid illness can manifest itself as hypothyroidism. Female patients are more likely to develop hypothyroidism [1].

The conditions that thyroid disease causes are very similar to other diseases, so distinguishing is sometimes difficult. Another type of hormone produced is called calcitonin. An appropriate amount of iodine is essential for the gland to produce these hormones.

Because it produces hormones, the thyroid gland impacts the human body's metabolic processes. An increase in thyroid hormone production causes hyperthyroidism. The use of an online ensemble of decision trees to detect thyroid-related disorders is proposed in this research. This study is aimed at increasing thyroid illness diagnosis accuracy [2].

Thyroid dysfunction is a classification problem and can be solved using data mining techniques. The symptoms of thyroid disease include high cholesterol, high blood pressure, and an unusual pulse rate. Using data analysis for thyroid disease classification, we can make data-based decisions to diagnose this disease on time accurately.

In the recent decade, disorders of the human body's glands have developed alarmingly. The thyroid is one of these glands whose sickness has spread worldwide. The thyroid gland's primary job is to check metabolism and cell activity [3].

Our model will help medical professionals to predict and use this classifier for further study and diagnosis. So the primary purpose of this research is to use a machine learning algorithm to diagnose thyroid dysfunction.

The crucial and difficult work in the healthcare profession is to detect health concerns and provide adequate treatment of disease at an early stage. There are certain disorders that can be recognized and treated early [4]. Based on the classification, Data mining is used in various healthcare services.

Based on the classification, machine learning is used in various medical services. The most important and difficult responsibility in the medical industry is to diagnose a patient's health problems and give proper care and treatment for the disease early. As an example, consider thyroid illness. Thyroid diagnosis is traditionally done by a comprehensive examination and numerous blood testing [5].

Thyroids are helpful to the overall body. Its probable failure might result in thyroid hormone production that is either inadequate or excessive. As a result of one or more swellings growing inside the thyroid, it might become inflamed or enlarged. Some of these nodules may harbour cancerous tumors. Sodium levothyroxine, often known as LT4, is a synthetic thyroid hormone used to treat hypothyroidism [6].

## 2. Literature Review

Few studies have been performed on thyroid disease, and the authors have evaluated many of the studies to create a proper background on the disease classification. Gou and Du proposed a system [7] that consists of a Generalized Discriminant Analysis and Wavelet Support Vector Machine System (GDA_WSVM) approach for the analysis of thyroid illnesses which incorporates three phases. Yang et al.'s targets are diagnosing thyroid illnesses with a professional system [8]. These are feature extraction – feature reduction phase, classification phase, and test of GDA_WSVM for correct diagnosis of thyroid diseases phase.

In the proposed system, fuzzy regulations are incorporated via the fuzzy neuron technique.

Poudel et al. [9] proposed that information benefit primarily based on a synthetic immune popularity system (IG-AIRS) might help diagnose thyroid characteristics primarily based totally on laboratory tests and might open the manner to numerous unwell diagnoses aided by the use of the latest scientific exam data. Parkavi centred on ant primarily based clustering algorithms. The category used distinct dissimilarity metrics like Euclidean, cosine, and Gower measures. The category used is distance primarily based category systems.

Prerana et al. used digital biosignal devices to determine thyroid dysfunction and used AI/Ml to distinguish between benign and malignant thyroid disease [10]. In [11], the authors used the local Fisher discriminant analysis (LFDA) and kernelized extreme learning machine method for thyroid disease diagnosis. Shankar et al. [12] evaluated the TUSP automated detection technique to predict thyroid disease by removing the long ultrasound imaging process. Aswathi and Antony [13] used unlabeled data to perform unsupervised learning to improve thyroid classification problems and optimize them. In [14], the CNN is evaluated to detect thyroid disease by using ultrasound images to improve the accuracy of the disease's prediction.

Banu [15] has targeted growing an AIS-based device gaining knowledge of a classifier for clinical analysis and investigating the functionality of the proposed classifier. The proposed classifier efficiently advanced the identity manner of thyroid gland disease.

The goal of Senashova and Samuels [16] is to create a professional gadget for thyroid prognosis. In [17], an expert system for thyroid disease diagnosis (ESTDD) is used. In this professional gadget, authors have used neuro-fuzzy regulations that can diagnose thyroid illnesses with 90.33% accuracy. In [18], Kang et al. used machine models to classify the dataset and improve the classification precision by 10% by dataset manipulation. The authors in [19] used the particle swarm optimization technique to enhance the feature selection process in disease detection. Han et al. used a Bethesda technique to detect thyroid nodules in patients in the Brazilian thyroid centre [20]. An LDA technique was presented in [21] that used the feature extraction method to increase the accuracy of the thyroid disease prediction model.

Automatic and precise thyroid nodule detection in ultrasound pictures is critical for reducing effort and radiologists' mistake rate. Even though deep learning has demonstrated high image classification performance, the intrinsic restrictions of medical pictures, such as a small dataset and time-consuming access to lesion labels, pose hurdles to this effort [22].

On pathological image classification benchmarks, deep learning approaches have shown promise. However, few studies on thyroid cancer autoclassification have been conducted due to the intricacy of pathological thyroid carcinoma pictures and labeled data's paucity [23].

## 3. Proposed Methodology

The proposed framework will take input in the form of dataset and then forward to the preprocessing module. In the preprocessing module, the normalization of images is performed in this module. After preprocessing the images, augmentation is performed. In augmentation, the dataset is divided into two parts: the training dataset and the testing dataset. After the augmentation process, import AlexNet and compare it with the customized AlexNet, and meet the criteria and store it in a trained model as shown in Figure 1. The missing values will be checked in the preprocessing steps. If we detect a missing value, the mean value will replace the value in that column. As the missing value had a data loss of about 91%, that parameter is removed from the dataset. We have adapted the dataset to be better processed with the chosen models. Initially, only two columns are removed. In the second step of the methodology, we performed dataset manipulation by undersampling the classes. Classes 0 and 1 are highly different in size: class 0 has 2870 samples, while class 1 only contains 293 values. The uneven class representation will cause the accuracy to be very high as machine learning algorithms are sensitive to skewed values. The results will contain many false-positive values, and accuracies will be high compared to the more balanced dataset as shown in Figure 2.

The last step was to divide the dataset into training and testing datasets. We have kept the traditional spill which is 70 percent of the data used for the training and 30 percent of the dataset used for testing purposes. While keeping in mind the dataset distribution, we have to oversample the majority class (class 0) and undersample the minority class (class 1).

Extracting accurate information for medical purposes is an essential task, and it defiantly helps future medical decisions. Feature selection is made to reduce the dimensionality in the dataset. It removes the irrelevant and redundant entries in the dataset. Hence, it increases the accuracy and improves the results. The feature selection identifies the most relevant features for the classification in the classification problems. When raw data is extracted many times, there are missing values in the dataset. The primary demographics contain information regarding the diseased patient's age, gender, medication, patient condition, and hormone levels like TSH, T3, and TT4 and category. The classification will contain two classes. Class 0 is negative, and class 1 is positive. Normal means that the patient is not suffering from thyroid disease.

### 3.1. Preprocessing Steps

1. Data cleansing
2. Data processing
3. Data elimination
4. Data wrangling

Preprocessing is arranged to overcome the different processing issues involving noisy data, redundant information, and missing values. The high quality of data will produce high-quality results according to the measuring metrics. The cost of computations will also reduce.

## 4. Simulation Environment

The experiments will be performed on a machine Core i5, with 8 GB RAM 500 hard disks. The programming language used is Python 3. The backend is based on Anaconda and Jupyter Notebook. We are utilizing Jupyter Notebook as it will provide the benefits of running on the online servers as shown in Table 1.

The *K*-nearest neighbor is a simple supervised machine learning algorithm; it is mostly used for the classification and regression problem. The model classifies the data on the points which are most similar to it. It classifies basically on the similarity measure as shown in

(1) $$\begin{array}{c} d\left(x,y\right)=\sqrt{\overset{m}{\underset{i=1}{\sum }}\;{\left(x_{i}-y_{i}\right)}^{2}}. \end{array}$$

Biological neural networks inspire ANN. It is a collection of nodes called neurons. It simulates the behaviour of biological systems. ANN can be used in both supervised and unsupervised training. A node receives the input from an external source in the form of a pattern interpreted, and output is created in equations (2) and (3).

(2) $$\begin{array}{c} \;z=f\left(b+x\cdot w\right)=f\left(b+\overset{n}{\underset{i=1}{\sum }}\;x_{i}w_{i}\right)x\in d_{1\times n},w\in d_{n\times 1},b\in d_{1\times 1},z\in d_{1\times 1}. \end{array}$$

Naïve Bayes is a very proficient and scalable algorithm. It is based on the Bayes theorem. Naïve Bayes is used in many data mining problems.

(3) $$\begin{array}{c} P\left(y\;|\;X\right)=\frac{P\left(X\;|\;y\right)P\left(y\right)}{P\left(X\right)}. \end{array}$$

Random forest contains decision tree classifiers. Randomly sample a subset of the training set to train each tree, and then, a decision tree is built. Random forest resolves the issue of overfitting in the training set; that is why it is preferred over the decision tree.

(4) $$\begin{array}{c} \text{RF}fi_{i}=\frac{\sum_{j}\;\mathrm{norm}\;fi_{ij}}{\sum_{j\in \text{all features},k\in \text{all trees }}\;\mathrm{norm}\;fi_{jk}}. \end{array}$$

The dataset is obtained from the UCI data thyroid disease repository. It includes 7200 multivariate types of records. Each record has 25 features. 18 are continuous data types, and 7 are discrete data types as shown in Table 2.

In addition to the upper description, the classes are subdivided as follows:

- Class 0: negative—2870 samples
- Class 1: positive—293 samples

The dataset contains missing values represented in Figure 3, with a question mark. Remove those features to reduce the data loss. With this step, we will achieve better accuracy after the classification. From the above, we can evaluate that the dataset is imbalanced with more negative occurrence than positive. So, class 0 is the majority class. When the dataset is imbalanced, it requires sampling to equalize the dataset and make the class representation equal to get better accuracy.

The proposed thyroid classification algorithm (Algorithm 1) takes the input from the dataset and performs a number of steps to identify the best classifier for the thyroid disease dataset.

The dataset was downsampled as shown in Figure 4 to make the classes equal in both cases. As the machine learning models are sensitive to skewed data, we equalized the dataset; therefore, our results will be accurate rather than paradoxical.

In Figure 4, the dataset has been acquired through the UCI dataset thyroid disease repository, and focus on implementing it on machine learning algorithms. The dataset contains the attributes of age, gender, and some thyroid markers like TSH, T3, and T4U to categorize the disease.

After dataset analysis, we determined that only a minority of the cases in the dataset are positive for the disease. In Figure 5, TSH, FTI, and T3 measurements are adding all the value to classify the model; they add up to 90% towards the classification as these features contribute more to the dataset alone as shown in Table 3.

The performance is evaluated based on different statistical measures, and sensitivity, specificity, precision, and recall were utilized to measure the results of the machine learning algorithms [24, 25]. The true positive rate refers to the accurately classified positive classes in the machine learning model as shown in

(5) $$\begin{array}{c} \text{True Positive Rate}=\frac{\text{ True Positive }}{\text{ False Negative}+\text{True Positive }}. \end{array}$$

The data points correctly classified as negative and originally negative are considered true negative rates in

(6) $$\begin{array}{c} \text{True Negative Rate}=\frac{\text{ True Negative }}{\text{ True Negative}+\text{False Positive }}. \end{array}$$

Precision is a good indicator of the accuracy of a model. It measures how many times a positive class is encountered during the testing phase. The precision will explain the classifier's accuracy and display actual positive values in the results as shown in

(7) $$\begin{array}{c} \text{Precision}=\frac{\text{ True Positives }}{\text{ True Positives}+\text{False Positives }}. \end{array}$$

Recall calculates how many times the model labeled a positive value true positive as shown in

(8) $$\begin{array}{c} \text{Precision}=\frac{\text{ True Positives }}{\text{ True Positives}+\text{False Negatives }}. \end{array}$$

*F*1 score is a harmonic mean between precision and recall and cannot avoid the other measure of *F*1, which is a function of precision and recall. The greater the *F*1 score, the higher the model's performance in

(9) $$\begin{array}{c} F1=2*\frac{1}{\left(1/\text{precision }\right)+\left(1/\text{recall }\right)}. \end{array}$$

A score is needed to balance between precision and recall.

## 5. Experimental Results and Analysis

After the implementation of the algorithm, we conducted a comparison of all the classifier results [13, 26]. We evaluated the results based on the true positive and true negative rates. True positive rates are the patients who do have the disease, and true negative rates are those who do not have the disease.

This proposed system is evaluated in the comparative results based on whether the person has the disease or not. Sensitivity and specificity are used to display the results. KNN [27, 28] is the least impressive model that can be used to classify the disease. It produced 59% and 91% specificity results. On the other hand, random forest produced the best results with 94.8% and 91% on the dataset. Naïve Bayes performed at 93% and 78%, and ANN produced 94% and 81%, respectively, as shown in Table 4.

In the neighbors' classifier, two tests are carried out with the said model. The first consists of training and validating using the unbalanced database and partitioning the data, taking 30% for validation and 70% for training; the results are shown in Figure 6.

KNN result at different *K* values is shown in Table 5 with a sensitivity value of 99.7% when *K* = 20.

In the next phase, we sampled the classes and reduced the dataset's size to implement the KNN classifier. We are only taking 300 values of each class 0 and 1 to reduce the paradoxical accuracy. The results are shown in Table 6 with KNN result of 91% with a dataset.

The accuracy is less, but it contains more true positives and more true negatives. Due to the missing values and skewness in the dataset, the results with the unsampled dataset were high, but they contained many false positives and false negatives. While performing the artificial neural network (ANN) [29, 30], we utilized a 40 : 60 ratio of the dataset for training and testing. Firstly, implementation is performed on the unsampled dataset. The model is trained for 1000 epochs as shown in Table 7.

Next, we implemented the artificial neural network on an undersampled dataset with equal class representation in both scenarios. Both the positive and negative values were set to 300 to improve the accuracy of the results.

For the third experimentation, we are using a random forest classifier. We are using 30/70 percent data split for the training. The number of estimators is 15, as shown in Table 8.

Next, we implemented the model on a downsampled dataset that contains equal values of both classes. The numbers of trees in the forest are 100, at which we drew our conclusion of the results as shown in Table 9.

In the last, we implemented the naïve Bayes algorithm on both the unsampled and sampled datasets. The results are discussed in Table 10.

The naïve Bayes algorithm is applied on a downsampled dataset of 300 values of each class. The conclusion is drawn after 20 k-fold cross-validations in Table 11.

## 6. Overall Result System

Compared to the overall results with four classifiers on the same dataset, KNN and random forest showed better results with 94.8% system accuracy.

## 7. Conclusion

This study signifies machine learning and data mining techniques to benefit the medical field and healthcare system. According to the regular protocol, this study will help the doctors use this as a supplementary system. We have evaluated the dataset based on precision and recall. Random forest was performed to be 94.8 percent accurate on average. Random forest is the most efficient in classification, and KNN is the least efficient.

On the other hand, ANN and naïve Bayes performed a level above the average of the KNN. With more training and a more extensive dataset, as expected, there will be better results from the artificial neural network. Our proposed method may also be helpful in creating a medical-related application or use it with neuro-fuzzy interference. The efficient and accurate diagnosis of thyroid disease will benefit the whole medical community. The healthcare system can be further enhanced, and better medical decisions can be taken.

## Figures and Tables

**Figure 1:** Proposed framework.

**Figure 2:** System diagram.

**Figure 3:** Dataset distribution.

**Figure 4:** Downsampled dataset.

**Figure 5:** Features contributing to classification.

**Figure 6:** Classifiers' performance.

**Algorithm 1:** Thyroid disease classification algorithm.

**Table 1:** Machine specification for simulations.

Specifications	Value
CPU	1.5–2.7 GHZ
GPU	920 m NVidia
RAM	12 GB
Generation	4^th^
Internet	8 Mbps upload, 8 Mbps download

**Table 2:** Dataset description.

Dataset characteristics	Multivariate, domain theory	Number of instances	7200	Area	Life
Attribute characteristics	Categorical, real	Number of attributes	25	Date donated	1987-01-01
Associated tasks	Classification	Missing values?	N/A	Some web hits	254314

**Table 3:** Dataset attributes.

Attribute	Value
Age	Integer
On thyroxine	Male (M), female(F)
Query on thyroxine	False (f), true (t)
On antithyroid	False (f), true (t)
Sick	False (f), true (t)
Pregnant	False (f), true (t)
Thyroid surgery	False (f), true (t)
T131 treatment	False (f), true (t)
Query hypothyroid	False (f), true (t)
Query hyperthyroid	False (f), true (t)
Lithium	False (f), true (t)
Goiter	False (f), true (t)
Tumor	False (f), true (t)
Hypopituitary	False (f), true (t)
Psych	False (f), true (t)
TSH measured	False (f), true (t)
TSH	Real
T3 measured	False (f), true (t)
T3	Real
TT4 measured	False (f), true (t)
TT4	Real
T4U measured	False (f), true (t)
T4U	Real
FTI measured	False (f), true (t)
FTI	Real
TBG measured	False (f), true (t)
TBG	Real
Referral source	SVHC, other, SVI, STMW, SVHD
Class	Negative (1), positive (0)

**Table 4:** Comparison of all classifiers.

Classifier	Sensitivity	Specificity
(1) KNN	59%	91%
(2) ANN	94%	81%
(3) Naïve Bayes	93%	78%
(4) Random forest	94.8%	91%

**Table 5:** KNN result at different *K* values.

*K*	Train	Sensitivity	Specificity
2	93.7%	99.1%	0.11
10	92.6%	99.5%	0.05
20	92%	99.7%	0.08
25	91.8%	99.6%	0.009

**Table 6:** KNN result with a sampled dataset.

*K*	Sensitivity	Specificity
2	67%	80%
10	70%	89%
20	65%	91%
25	59%	91%

**Table 7:** ANN result with 1000 epochs.

Epochs	Sensitivity	Specificity
1000	77.4%	99%

**Table 8:** Random forest result.

Classifier	Sensitivity	Specificity
Random forest	84.4%	99.4%

**Table 9:** Random forest result.

Classifier	Sensitivity	Specificity
Random forest	94.8%	91.2%

**Table 10:** Naive Bayes result.

Classifier	Sensitivity	Specificity
Naïve Bayes	98%	97%

**Table 11:** Naïve Bayes result.

Classifier	Sensitivity	Specificity
Naïve Bayes	93%	78%

## Data Availability

Data can be available upon request.
